RETRACTED

# Growth inhibition and apoptosis in colorectal cancer cells induced by Vitamin D-Nanoemulsion (NVD): involvement of Wnt/β-catenin and other signal transduction pathways

**DOI:** 10.1186/s13578-019-0277-z

**Published:** 2019-02-01

**Authors:** Suhail Razak, Tayyaba Afsar, Ali Almajwal, Iftikhar Alam, Sarwat Jahan

**Affiliations:** 1 Department of Animal Sciences, Faculty of Biological Sciences, Quaid-i-Azam University, Islamabad, Pakistan; 2 Department of Community Health Sciences, College of Applied Medical Sciences, King Saud University, Riyadh, Kingdom of Saudi Arabia

**Keywords:** Vitamin D, CRC, Wnt/β-catenin, Cell cycle, NVD

## Abstract

**Background:**

More than the two decades, the question of whether vitamin D has a role in cancer frequency, development, and death has been premeditated in detail. Colorectal, breast, and prostate cancers have been a scrupulous spot of center, altogether, these three malignancies report for approximately 35% of cancer cases and 20% of cancer demises in the United States, and as such are a chief public health apprehension. The aim was to evaluate antitumor activity of Vitamin D-Nanoemulsion (NVD) in colorectal cancer cell lines and HCT116 xenograft model in a comprehensive approach.

**Methods:**

Two human colorectal cancer cell lines HCT116 and HT29 (gained from College of Pharmacy, King Saud University, KSA were grown. 3-(4, 5-dimethylthiazol-2-yl)-2, 5-diphenyl tetrazoliumbromide protocol were performed to show the impact of NVD and β-catenin inhibitor (FH535) on the viability of HCT116 and HT29 cell lines. Apoptosis/cell cycle assay was performed. Analysis was done with a FACScan (Becton–Dickinson, NJ). About 10,000 cells per sample were harvested and Histograms of DNA were analyzed with ModiFitLT software (verity Software House, ME, USA). Western blotting and RT-PCR were performed for protein and gene expression respectively in in vitro and in vivo.

**Results:**

We found that NVD induced cytotoxicity in colorectal cells in a dose-dependent manner and time dependent approach. Further, our data validated that NVD administration of human colorectal cancer HCT116 and HT29 cells resulted in cell growth arrest, alteration in molecules regulating cell cycle operative in the G2 phase of the cell cycle and apoptosis in a dose dependent approach. Further our results concluded that NVD administration decreases expression of β-*catenin* gene*, AKT* gene *and Survivin* gene and protein expression in in vitro and in vivo.

**Conclusion:**

Our findings suggest that targeting β-catenin gene may encourage the alterations of cell cycle and cell cycle regulators. Wnt/*β*-*catenin* signaling pathway possibly takes part in the genesis and progression of colorectal cancer cells through regulating cell cycle and the expression of cell cycle regulators.

RETRACTED

**Electronic supplementary material:**

The online version of this article (10.1186/s13578-019-0277-z) contains supplementary material, which is available to authorized users.

## Introduction

Colorectal cancer (CRC) is an all-inclusive problem with a yearly frequency of roughly 1 million reports and a yearly death of more than 100,000 [1, 2]. The utter number of cases will rise over the subsequently 2 decades as a consequence of aging and growth of populations all over countries. The danger for this malignancy differs from region to region and/or inside countries. The jeopardy also fluctuates among individual people depend on diet, lifestyle, and genetic factors. In Europe, Colorectal cancer (CRC) is the second main public cancer and subsequent foremost source of cancer death after lung cancer, with an approximated overall frequency of 447 per 100,000 [3, 4]. 1,25(OH)_2_ D_3_ interferes with numerous signaling pathways, which could partly intercede its antitumoral activity. Various observations have illustrated that 1,25(OH)_2_D_3_ hampers the WNT/β -catenin pathway and the commencement of its candidate genes in colorectal cancer cells, which play a crucial part in inhibition of cell propagation and upholding of the distinguished phenotype [5, 6]. 1, 25(OH)_2_D_3_ hampers the WNT/β-catenin pathway via numerous mechanisms. Primary, it swiftly raises the sum of Vitamin D receptor (VDR) attached to β-catenin, therefore tumbling the association involving β-catenin and the transcription factors of the TCF/LEF family. Thus resulting to the suppression of its candidate genes [5]. An observation demonstrated the VDR/β-catenin association and exemplified the involved protein domains. Whereas another study illustrated that wildtype APC boosts the reticence of β-catenin/TCF transcriptional effect by 1,25(OH)_2_D_3_ [7, 8]. Subsequently, 1,25(OH)_2_D_3_ persuades β -catenin nuclear export allied to E-cadherin increase at the plasma membrane adherent junctions [5]. Lastly, it persuades the expression of DKK1, an extracellular WNT inhibitor [9]. Besides that, 1,25(OH)_2_D_3_ hampers the creation of IL1β by THP-1 monocytic leukemia cells and, if extrapolated to tumor-allied macrophages, this would symbolize one more mechanism of prevention of β-catenin/TCF-dependent gene commencement in CRC cells, as IL1 β hampers β-catenin phosphorylation and tagging for deprivation by GSK-3 β [10]. Therefore, 1,25(OH)_2_D_3_ applies a composite set of dogmatic activities resulting in the prevention of the WNT/β-catenin pathway. Since this pathway is deviantly triggered in most adenomas and colorectal tumors and is known as the chief element in this neoplasia, its reticence is doubtless critical for the anti-tumoral activity of 1,25(OH)_2_D_3_ in CRC. Moreover, 1,25(OH)_2_D_3_ sensitizes CRC cells to the growth inhibitory activity of TGF-β by up-regulating the expression of its type I receptor (TGFBR1) [11]. Furthermore, 1,25(OH)_2_D_3_ hampers the stimulation of cell propagation by Epidermal growth factor (EGF) through the attenuation of EGF receptor (EGFR) expression and the stimulation of its internalization after ligand binding [12]. 1,25(OH)_2_D_3_ may also hamper EGFR action by enhancing the expression of E-cadherin [5] and by suppressing that of SPROUTY-2 [13], which are uncooperative and confirmatory regulators of EGFR effect, respectively [14, 15]. Similarly, 1,25(OH)_2_D_3_ hinder the growth-stimulatory activity of insulin growth factor 2 (IGF2) via the inhibition of IGF2 discharge and the enunciation of the expression of various genes encoding IGF-binding proteins (IGFBP) [16, 17].

RETRACTED

In spite of frequent studies suggesting the cytotoxicity of 1, 25(OH)_2_D_3_ in countless cancer cell lines, the mechanism of action of the 1,25(OH)_2_D_3_ throughout tumor decline is predominantly veiled. Consequently, our study, investigated the anticancer properties of vitamin D-Nano-emulsion (NVD) in an efficient approach, using in vitro and in vivo model systems. It was seen that NVD encourages frequent fold advanced intensity of cytotoxicity in malignancy. Auxiliary, we showed growth obstruction and initiation of apoptosis in CRC cells encouraged by NVD, down regulation of Wnt/*β*-*catenin* signal transduction pathway, Anti-proliferative effect of administration of NVD, β-catenin Inhibitor (FH535) in HCT116 and HT29 cells, Flow cytometric analysis of colorectal cancer cells after NVD treatment for apoptosis and cell cycle, Inhibition of colony formation in HCT116 and HT29 cells after administration with NVD and amendment in CTNNB1 protein intensity after NVD administration. Therefore our data specify that NVD may possibly be developed further as a prospective anti-cancer agent, both in conventional and combination therapy.

## Materials and methods

### Ethical declaration

Athymic nude mice studies were carried out according to the Institutional principles for the concern and use of animals. The experimental protocol was approved (BAS#0256) by the ethical board of Quaid-i-Azam University, Islamabad, Pakistan and College of Pharmacy (Committee dealing animal care and use), King Saud University, Riyadh, KSA. Before onset of the experiment on human colorectal cancer cell lines HCT116 and HT29 (ATCC^®^ CCL-247 ™ and ATCC^®^ HTB-38 ™ respectively) purchased in July 2017 from American Type Culture Collection (MD, USA), ethical approval was taken from ethics committee of preclinical studies, college of Pharmacy, King Saud University, KSA.

RETRACTED

### Cell culture

Two human colorectal cancer cell lines HCT116 and HT29 (obtained from College of Pharmacy, King Saud University, KSA) were cultured in a 5% CO_2_ atmosphere at 37 °C in medium containing Dulbecco’s Modified Eagle’s Medium (DMEM) (ATCC^®^ 30–2002™), 10% fetal bovine serum (FBS, Gibco) as well as 1% penicillin/streptomycin. NVD and β-catenin inhibitor (FH535) dissolved in DMSO was applied for cell treatment. Cells with 70% confluency were induced with NVD and β-catenin inhibitor at 10–100 µM for 48 h in cell culture medium and the dilution of DMSO applied for each treatment was 0.1% (V/V).

### Cell viability assay/MMT assay

3-(4, 5-dimethylthiazol-2-yl)-2, 5-diphenyl tetrazoliumbromide protocol was carried out to show the effect of NVD and β-catenin inhibitor (FH535) on the viability of HCT116 and HT29 cell lines. The cells were plated (1 × 10^4^ cells per well) in 1 ml of culture medium consisting of 10–200 µM dilution of in 24-well microtiter plates. Cells were kept in a humidified incubator for 48 h at 37 °C, 200 µl of 3-94,5-dimethylthiazol-2-yl)-2,5-diphenyl tetrazoliumbromide (5 mg/ml phosphate buffer saline, PBS) was supplemented to each well and kept for 2 h, 200 µl of DMSO was added to each plate which was then spun (1800 × g for 5 min at 4 °C). The readings at 540 nm wavelength were noted on a microplate reader (Elx 800). Impact of NVD and FH535 β-catenin inhibitor on inhibition of growth was calculated as  % cell viability as DMSO-treated cells were kept as control. Absorbance numbers of media containing wells were subtracted from test sample values.

$${\text{Cell}}\,{\text{viability}} = \left[ {\frac{{{\text{Absorbance}}\,{\text{of}}\,{\text{Sample}} - {\text{Absorbance}}\,{\text{of}}\,{\text{Blank}}}}{{{\text{Absorbance}}\,{\text{of}}\,{\text{DMSO}} - {\text{Absorbance}}\,{\text{of}}\,{\text{Blank}}}}} \right] \times 100$$

HCT116 cells and HT29 cells were collected consequently to treatments with active NVD for 48 h. Cells were suspended in a fresh medium, cell number was determined, and 500 cells (HCT116) or 1000 cells (HT29) were plated in triplicate into 35 mm cell culture dishes. After 7 days in culture, colonies were stained with 0.5% crystal violet as described [18]. Cell colonies were counted under dark field using a cubic colony counter (AO scientific). The number of cells in each colony was determined by phase contrast microscopy, and colony sizes were measured on images using Adobe Photoshop software. Data was represented as colony number in NVD group relative to expressed as mean ± SEM of three separate tests.

RETRACTED

#### Cell cycle analysis

All HCT116 and HT29 were administrated with NVD (20–60 µM, 48 h) in inclusive medium were trypsinized. Then fixed in 1% paraformaldehyde:1xpbs. Then washed twice with cold PBS and spun. Chilled 70% ethanol was used to suspend cell pellet and incubated overnight. The cells were spun for 5 min at 1000 rpm and the pellet obtained was washed twice with Chilled PBS to remove ethanol then finally cells are labeled with FITC and propidium iodide (PI) using the Apo-Direct Kit (BD Pharmagen, CA). the analysis was done with a FACScan (Becton–Dickinson, NJ). About 10,000 cells per sample were harvested and Histograms of DNA were analyzed with ModiFitLT software (Verity Software House, ME, USA).

### Extraction of protein and Western blot analysis

SDS-PAGE and western blot investigations were performed by previously developed protocol with slight modifications [19, 20]. Briefly, after 24 h, and 48 h of treatments with NVD at vital doses, HCT116 and HT29 cells were lysed in DMEM augmented with freshly added protease and phosphatase inhibitor cocktail 1:100 (Santa Cruz, CA) and protein concentration were estimated by Bradford assay [21]. For western blotting 8–12% polyacrylamide gels were used to resolve 40 μM of protein, transferred on to a nitrocellulose membrane, probed with appropriate monoclonal primary antibodies, and detected by super signal west Pico, Dura or Femto Chemiluminescence Reagent (Thermo Scientific, USA). Quantification of protein bands was done through measuring band density using Image J software. The densities of the bands (normalized to actin) relative to that of the untreated control (designated as 1.00) were presented as mean ± SEM of three separate experiments.

### Gene expression analysis

Whole RNA was extracted (RNeasy Mini Kit (Cat No./ID: 74104) from the cells using the following method. RNA dilution was determined by using a spectrophotometer at 260 NM and cDNA was prepared by following the manufacturer protocol (BioLabs E6300) using the kit. The reaction mixture was prepared containing 10 µl FastStart Universal SYBR Green Master (Roche, Germany), 6 µM reverse primers, and 10 µg cDNA, with RNAase free water added to a total volume of 20 µl. The amplification and real time analysis were done for 40 cycles with following factors; 95 °C (10 min) in order to activate of FastStart Taq DNA polymerase; 60 °C (1 min) for amplification and real-time analysis. The gene expression levels were determined using 2^−ΔΔCT^. Primer sequences used were;

*CTNNB1* Sense 5ʹ-TGTGAATCCCAAGTACCAGTGT-3ʹ

*CTNNB1* Antisense 5ʹ-CGTCAGACAAGGAGAAACATT-3ʹ

*β*-*Actin* Sense 5ʹ-CCTCTTCCTCAATCTCGCTC-3ʹ

*β*-*Actin* Antisense 5ʹ-GCTCAATGTCAAGGCAGGAG-3ʹ

RETRACTED

### Imunofluorescence microscopy

HCT116 and HT29 cells were cultured in a two chamber tissue culture glass slides and were administrated with 40 µM of NVD at 75% confluence for 24 h. Once the chamber was removed, Phosphate buffer was used to rinse the slides, 2% paraformaldehyde was used to fix the cells and permeablized in methanol. Slides were rinsed with phosphate buffer and 2% serum was used as a blocking agent. Incubation with primary antibody overnight was followed by incubation with appropriate fluorophore-tagged secondary antibody. For mounting antifade 4, 6-diamidino-2-phenylindole, dihydrochloride (DAPI) (invitrogen NY) was used to apply and hematoxylin for counter staining. The analysis was done by using Bio-Rad Radiance system (2100 MP Rainbow) for imaging at the college of pharmacy, King Saud University, KSA. To detect apoptotic and necrotic cells, the Annexin-V-fluos staining Kit (Roche, Switzerland) was used according to the kit’s procedure. Zeiss 410 confocal microscopy was used to measure fluorescence. Annexin V and propidium iodide were used to stain the cells. The unstained cells in a selected field were calculated to determine the level of necrosis as well as apoptosis.

### Development and characterization of pea protein-stabilized nanoemulsions and protein vitamin D-pectin nanocomplexes (NVD)

Pea protein (3 g) with 90% pea protein (dry basis) was added to 100 ml deionized water. Stirred for 30 min at room temperature (23 °C). Pea protein dispersion was adjusted to pH 12 with 2 M NaOH. Ultrasound was applied using a laboratory scale mano-thermo-sonication (MTS) system. A VC-750 ultrasound generator at 20 kHz (Sonics & Materials) was used to deliver acoustic energy to a probe (12.5 mm diameter) placed in a specially designed sonoreactor. Different ultrasound techniques will be applied after pH-shifting to pH 12 for 1–5 min, including manosonication (MS), thermosonication (TS), and mano-thermosonication (MTS). After ultrasound treatment, samples were held 1 h (room temp) prior to the adjustment to pH 7 with 2 M HCl. Protein dispersion without treatment was served as the control. Neutralized protein dispersions were centrifuged (1200*g*, 15 min, 20 °C). Supernatants were collected for further analyses, including protein content, mean particle size (d_32_ and d_43_), and sodium dodecyl sulfate polyacrylamide gel electrophoresis (SDS-PAGE).

Nano-emulsions were prepared with vitamin D (VD) and pea protein modified with above-mentioned methods as an emulsifier. VD concentrations are 0.5, 1.0, and 2.0% (v/v) in the nano-emulsions. A set dose of soluble pea protein (2.0%, w/v) was utilized. The VD and soluble pea protein were assorted (5 min), followed by sonication (1–5 min) and/or homogenizing by IKA Labor Pilot colloidal mill to obtain the nanoemulsion. Pectin (0.01–0.5%, w/v) was added to nanoemulsion as a stabilizer. Nanoemulsion without pectin was prepared as a control. Pea protein–VD-pectin nanocomplexes were prepared at different protein: VD ratios. VD was slowly added to soluble pea protein with strong stirring at the determined optimum protein to VD molar ratios. The pH values of the nanoemulsion and nanocomplex pH was accustomed from 3 to 7. Particle size (d_32_ and d_43_) and stability of the nanoemulsions and nanocomplexes were calculated. Centrifugation was done to measure the Physical stability of nanoemulsions.

RETRACTED

### In vivo tumor xenograft model

Athymic male mice were acquired from King Faisal Hospital and research center, Riyadh, KSA, were homed under contamination free environment (12 h day/12 h night schedule), and nourished with a sterilized food adlibitum. HCT116 cells were selected for evaluating the in vivo impact of NVD and β-catenin inhibitor (FH535) as they generate fast tumors in mice. Cells were harvested, suspended in complete DMEM. Tumor xenografts HCT116 cells in mice were established by injecting cells (1 × 10^6^) subcutaneously mixed with Matrigel (Collaborative Biomedical Products, Bedford, MA) in a ratio of 1:1.

Thirty mice were categorized into three groups.

- *Group1* Served as Control Group, consisting six mice, received DMSO intra-peritoneally (i.p).
- *Group2* Divided into two subgroups; Group 2a and 2b consisting of six animals each. Received NVD (15 and 25 mg/kg) intra-peritoneally (i.p) respectively, twice weekly.
- *Group3* Divided into two subgroups; Group 3a and 3b consisting of six animals each. Received FH535 (15 and 25 mg/kg) intra-peritoneally (i.p) respectively, twice weekly.

Throughout the study, body weight of animals, food and water expenditure were documented twice a week. Tumor volume was measured by digital caliper and calculated using the formula: L1 × L2 × H × 0.5238, where (L1 = long diameter L2 = short diameter and Height = height of the tumor).

Tumor sizes were recorded twice weekly. At the end of the experiment when tumor volume reached to ~ 1200 mm^3^ animals were sacrificed by CO_2_ inhalation was used as anesthesia. Tumors were resected, weighed and frozen at − 80 °C for subsequent western blotting, RNA extraction and immunohistochemistry.

### Immunohistochemistry

The immunohistochemistry was done by following the protocol described in our previous work [20].

RETRACTED

### Data analysis

Densitometry of western blot images was performed using an image analysis program (Image J 1.41; National Institutes of Health). Data of in vitro assays were analyzed GraphPad Prism 5 software to determine IC_50_ values. Level of significance between different treatments groups relative to control was estimated by oneway analysis of variance followed by Tukey’s multiple comparison tests. Comparison between more than one parameter was accomplished using two way analysis of variance (ANOVA) followed by Bonferroni multiple comparison test. *p* < 0.05 was considered statistically significant. Where required correlation analysis was done and R values were calculated.

## Results

### Vitamin D-Nanoemulsion (NVD) and FH535 inhibits growth and viability of colorectal cancer cells

To scrutinize the anti-proliferative prospective of NVD and FH535, we executed 3-(4, 5-dimethythiazol-2-yl)-2, 5-diphenyl tetrazolium bromide (MTT) assay against HCT116 and HT29 colorectal cancer cells. It was observed that NVD and FH535 treatment (0–100 μM for 24 h and 48 h) to CRC cells results in inhibition of cell growth in a concentration and time-dependent manner. Time course scrutiny revealed CRC cells respond to NVD and FH535 treatment within 48 h. The IC_50_ values of NVD and FH535 -treated HCT116 were 40.6 and 40.1 and 25.5 and 24.6 μM at 24 h and 48 h respectively while IC50 values of NVD and FH535 -treated HT29 cells were 50.1 and 43.5 at 24 h and 30.3 and 26.2 μM at 48 h (Fig. 1, Table 1). The data suggested that NVD and FH535 treatment showed a significant potential in inhibiting proliferation of HCT116 and HT29 cells.

**Fig. 1:** Inhibition of cell growth in colorectal cancer. 3-(4, 5-dimethythiazol-2-yl)-2, 5-diphenyl tetrazoliumbromide assay was carried out on two colorectal cancer cell lines HCT116 and HT29 cells in order to gauge the effect of NVD and FH535 administration on growth of these colorectal cancer cell lines ***P < 0.001 and **P < 0.01 vs. control.  % cell viability of HCT116 and HT29 cells were determined. Each value represents a mean ± SD (n = 3)

**Table 1:** IC 50 value of NVD against HCT 116 and HCT 29 cells in cell viability assay

Treatment	HCT 116		HCT 29	
	24 h	48 h	24 h	48 h
NVD (IC50 µM)	40.6	25.5	50.1	30.3
FH 535 (IC50 µM)	40.1	24.6	43.5	26.2

### Inhibition of clonogenecity in colorectal cancer cell lines

To conclude the consequence of NVD treatment on the clonogenicity of HCT116 and HT29 cells, clonogenicity assay was performed. HCT116 and HT29 cells were pre-treated with NVD at 40 and 60 µM doses substantiated a concentration dependent reticence of colonogenicity with deference to untreated control cells. Our results illustrate the clonogenicity of HCT116 and HT29 cells after treatment with NVD was patently condensed as compared to the control (Fig. 2).

RETRACTED

**Fig. 2:** Inhibition of cologenecity in colorectal cancer cells by NVD. (Clonogenic assay; 7 days). **a**, **b** NVD administration (40 and 60 μM) of HCT116 and HT29 cells inhibiting colony formation. Each value represents a mean ± SD (n = 3)

### Vitamin D-Nanoemulsion administration caused cell cycle arrest by flow cytometric analysis

To investigate whether NVD administration will cause the cell arrest, the flow cytometric analysis carried on HCT116 and HT29 cells administrated with NVD showed a noticeable dose- dependent boost of the cell population in the G2 state of the cell cycle. The G2-phase cell cycle distribution for HCT116 was 30.1% and 44.3% and for HT29 was 40.5%, and 48.3% at 40 and 60 µM doses of NVD respectively. This rise in the G2 state of the cell population was followed by a simultaneous decrease in the Go/G1 and S phase cell population (Fig. 3).

**Fig. 3:** **a**, **b** NVD treatment on HCT116 and HT29 cells resulted in accumulation of cells at the G2-phase and growth inhibition and apoptosis. After 24 h incubation of NVD treated cells and staining with propidium iodide, DNA content was analyzed by flow cytometry. **c**, **d** NVD treatment on HCT116 and HT29 cells resulted in accumulation of cells at the G2-phase. After 24 h incubation of NVD treated cells and staining with propidium iodide, DNA content was analyzed by flow cytometry. Percentage of cell population in G2-phase of the cell cycle is shown. Experiments were performed in triplicate

### NVD administration promotes apoptosis—flow cytometric Analysis

Apoptosis and cell cycle arrest are associated. To quantitatively examine whether NVD induces apoptosis of the HCT116 and HT29 cells, the analysis was performed by flow cytometry. Results showed a prominent concentration dependent boost in a population of dead cells, as a result of NVD treatment in HCT116 and HT29 cells. The percent apoptosis in HCT116 cells observed was 26.7% and 54% and for HT29 was 17.8% and 32.8% at a concentration of 40 and 60 μM of NVD respectively (Fig. 3, Table 2).

**Table 2:** Percentage of cell population after administration of NVD

NVD (µM)	% Apoptosis	
	HCT116	HT29
0	0.35 ± 0.02	1.92 ± 0.01
40	26.7 ± 0.03	17.8 ± 0.21
60	54 ± 0.14	32.8 ± 0.16

Mean ± SD of experiments performed in triplicate is shown

### Effect of NVD on the expression of cell cycle regulators, caspases and Bcl-2 family

To explore the molecular mechanisms of growth arrest induced by NVD, the cell cycle monitors were analyzed by western blotting for their expression levels. Results showed decreased protein expression of Cyclins A, B1, E2 and also decrease in Cdc25c levels after treatment of NVD in a dose-dependent manner in HCT116 and HT29. P21 showed increased expression levels (Fig. 4a, b).

RETRACTED

**Fig. 4:** Effect of NVD treatment of HCT116 and HT29 (**a**, **b**) cells on protein expression of cdc2, WAF1/p21, cdk 2, 4 cyclin A, B1, E2 and (**c**, **d**) showing active Caspase 3, 7, 9 and PARP. Cells were administrated with NVD (20, 40 and 60 μM) for 24 h and 48 h and harvested. Total cell lysates were prepared and 40 μM proteins was subjected to SDS page followed by immunoblot analysis and chemiluminescence detection. Equal loading of protein was verified by stripping the Immunoblot and again probing it for Actin. The immunoblots shown here are representative of three individual experiments with similar results

The expression levels of proteins allied to apoptosis were analyzed by immune- blotting. Pro-apoptotic proteins, Bak and Bax, demonstrated an increase in treated as well as in control. Apoptosis in HCT116 and HT293 cells was accompanied by loss of Bcl-xL protein expression, and results indicated that NVD induced noteworthy (*p* < 0.001) inhibition of Bcl-xL protein after 24 h of administration. The inhibitory effect of NVD against Bcl-2 protein expression was also decreased as like as Bcl-xL (Fig. 5a). In the NVD-administrated cells, the cleavage of PARP (Poly (ADP-ribose) polymerase and Caspases was measured. PARP is a crucial feature of early events in apoptosis and caspases are important proteases in mitochondria-mediated apoptosis. After treatment of NVD in HCT116 and HT29 cells for 24 h and 48 h, dose and time dependent cleavage of PARP (Poly (ADP-ribose) polymerase, caspase 7, 9 and 3 was observed. Enhanced cleavage of these proteins was seen at 48 h treatment. The enhanced cleavage appeared to correspond well with the increased apoptotic rate (Fig. 4c, d).

**Fig. 5:** **a** Effect of treatment of NVD to HCT116 and HT29 cell lines on protein expression of Bax, Bcl2, Bak and Bcl-X_L_. **b** Immunoblot analysis of β-catenin expression of HCT116 and HT29 in NVD treated group as compared to control group. The cells were administrated with NVD for 48 h and harvested and cell lysates prepared. The data are representative of three independent experiments with similar results

### NVD administration induces a decrease in β-catenin expression

Molecular, genetic and clinical data in humans are scant but they recommended that vitamin D is having a shielding effect against colon cancer [22]. Results showed a marked decrease in expression of the β-catenin protein in a concentration dependent approach on HCT116 and HT29 cells after administration with NVD (20, 40 and 60 uM) for 48 h by immunoblotting (Fig. 5b). To investigate whether the observed drop off in β-catenin protein was the consequence of diminished transcription of *β*-*catenin* gene, the mRNA expression of *β*-*catenin* gene was evaluated by administration of NVD in HCT116 and HT29 cells. A marked decrease was observed in mRNA expression in a dose dependent approach (Fig. 6a).

RETRACTED

**Fig. 6:** **a** Modulation of β -catenin expression by NVD treatment in HCT116 (**a**) and HT29 (**b**) cells. mRNA expression of β-catenin in NVD treated HCT116 and HT29 cells (RT-PCR), experiment performed in triplicate (mean ± SD), **p < 0.01. **b** Effect of NVD on protein expression of β-catenin, Survivin and phosphorylation of Akt at Ser473 in HCT116 and HT29 cells., Total cell lysate were prepared and 40 μM proteins was subjected to SDS-page followed by Immunoblot analysis and chemiluminescence detection. Equal loading of protein was confirmed by stripping the immunoblot and reprobing it for β-Actin

At a dose of 60 µM of NVD (treated), HCT116 and HT29 cells illustrated a decrease in β-catenin expression when compared with control (untreated) by immunofluorescence staining. Significant Alexa fluor staining of β-catenin (nucleus) of both cell lines (green fluorescence) (counter stain used was DAPI, blue fluorescence) was experiential in control, while the expression of β-catenin as specified by staining was noticeably decreased in NVD treated cells as shown in Fig. 7.

**Fig. 7:** Imunofluorescence staining of HCT116 (**b**) and HT29 (**d**) demonstrating expression of β-catenin in both NVD treated (60 µM) as compared to control HCT116 (**a**) and HT29 (**c**) cells (untreated). Alexa fluor staining of β-catenin of both cell lines (green fluorescence) and counter stained with DAPI (blue fluorescence) were observed

FH535 β-catenin inhibitor prevents survivin and Akt phosphorylation resulting down regulation of β-catenin protein expression. Compared with NVD treatment (60 μM), pre-incubation of HCT116 and HT29 cells with FH535 β-catenin inhibitor (20 μM) for 2 h before NVD treatment resulted in noteworthy decline in the protein expression of β-catenin, p-Akt, and survivin as observed by Immunoblot analysis (Fig. 6b).

### Signaling pathways and endurance proteins amended by NVD administration

Western blot analyses were executed to assess the consequence of NVD on signaling pathways engaged in cancer cell endurance and propagation. HCT116 and HT29 cells were administrated with 20, 40 and 60 µM of NVD. The effects of NVD on various signaling pathways in colorectal cancer cells were studied.

### NVD effect on CK2 and NFкB p65

Protein kinase CK2 (formerly referred to as casein kinase II) is an evolutionary conserved, highly pleiotropic, a ubiquitous protein kinase with multi- substrates controlling a wide range of cellular processes. CK2 α expression plays a crucial role in cellular as well as in organismal endurance. HCT116 and HT29 cells administrated with NVD for 24 h drastically diminished expression of the CK2α protein in a dose-dependent approach (Fig. 8a). Nuclear factor-κB (NF-κB) includes the family of transcription factors that play significant roles in inflammation, immunity, cell proliferation, differentiation, and survival. Aberrant NFκB regulation leads to constitutive cell survival by avoiding program cell death in various malignancies. Inducible NF-κB commencement depends on phosphorylation-induced proteasomal degradation of the inhibitor of NF-κB proteins (IκBs), which retain inactive NF-κB dimers in the cytosol in unstimulated cells.

RETRACTED

**Fig. 8:** Western blot analysis of cellular lysates prepared from HCT116 and HT29 cells. Lysates prepared from HCT116 and HT29 cells, initially seeded at density of 1.5 × 10^4^ cells were administrated with 20, 40 and 60 µM concentrations of NVD. The blots probed with CK2 αα’, PI3-K, STAT3, STAT P-Try705, NFκB p65 P-S529, IκBα P-S32/36 and xIAP antibodies were shown. Actin blots are shown as loading controls. Data based on three different experiments, each carried out in triplicate

In HCT116 and HT29 Cells administrated with NVD inhibited the expression of both NFкB p65 P-Ser529 and total NFκB p65 protein in a dose and time dependent approach. Moreover, protein expression of phospho-IκBα Ser32/Ser36 was significantly declined in a concentration and time dependent approach following NVD treatment (Fig. 8a, b).

### Impact of NVD on further signaling pathways

Numerous actions of the Ras/Raf/MEK/ERK and Ras/PI3-K/Akt/mTOR pathways on apoptosis are transitionally by ERK or Akt phosphorylation of key apoptotic effector molecules. The figure of ERK 1/2 phosphorylation targets are more than hundreds, thus suppression of MEK and ERK activities will have a reflective influence on cell growth. Results showed that NVD administration appreciably decreased phosphorylation of Akt and ERK1/2 in HCT116 and HT29 cells (Fig. 8b). The NVD administration on the expression of JAK-STAT signaling showed prominent loss of JAK2 protein expression in a time-dependent approach with a significant (*p* < 0.001) suppression of protein expression was exhibited after administration for 48 h. Prominent STAT3 has been allied with the growth, progression, and maintenance of many human tumors. Results showed that treatment with NVD for 48 h significantly declined phospho-STAT3 Tyr705. Also, NVD led to noteworthy inhibition of total STAT3 protein expression (Fig. 8a).

RETRACTED

### In vivo studies

#### NVD and FH535 β-catenin inhibitor administration results to momentous diminution in tumor volume

Colorectal cancer developed athymic (nu/nu) male nude mice were used for appraising antitumor effects of NVD. On the 8th day of injection of HCT116 cells, when an evident tumor was noticeable, nude mice were administered NVD (15 mg/kg and 25 mg/kg), intraperitoneally (i.p), twice weekly. The particular concentration of compound was chosen based on a pilot study. Result illustrated a notable diminution in tumor volume when administrated with NVD in contrast to untreated control animals bearing tumor after 15–17th day of administration. Though, the decrease in tumor size was more noteworthy in a case of 25 mg/kg NVD administrated mice.

#### Administration of NVD induce no toxicity in xenografts mice

No death was witnessed in NVD and FH535 treated (15 and 25 mg/kg) tumor bearing mice during the experimental period. Whilst untreated control nude mice survived for a maximum of only ~ 50 days, the NVD and FH535 administrated groups led to ~ fourfold amplification in the lifespan for at least 43% of mice. The organs from NVD and FH535 revealed no obvious variations in histo-architecture (Additional file 1). This corroborated that administration of NVD and FH535 results no side effects. Thus, our statistics illustrated that NVD and FH535 administration in nude mice decreases the tumor load, boost survival. On tumor section of control, NVD and FH535 administrated nude mice at 38th days of treatment, histopathology was carried out by hematoxylin and eosin staining (Fig. 9c).

**Fig. 9:** Consequence of NVD administration on HCT116 tumor growth in athymic nude mice. **a** Average tumor volume of water fed, 15 and 25 kg/mg NVD injected mice plotted over days after tumor cell inoculation. Values represent mean ± SD of six mice. *p < 0.01 (25 mg/kg); **p < 0.05 (15 mg/kg) vs water fed normal control mice ***p < 0.001. **b** The inhibition of xenograft tumor growth of human HCT116 by NVD and FH535 c) H&E staining of NVD administrated xenograft tumors (**b**) vs control (**c**)

In control tumor sections, high nuclear staining by hematoxylin revealed the presence of a large number of proliferating cells in contrast to treated tumor sections (Fig. 9c).

#### Caspases mediate confrontation to apoptosis by administration of NVD and FH535 in xenograft tumors

The result of NVD and FH535 on cleavage of Caspase 3 was reviewed sequentially to differentiate whether the growth inhibition of cells is due to the initiation of apoptosis (Fig. 10). The morphology of NVD and FH535administrated cells also illustrated support of cell death. Immunostaining of tumor sections from NVD and FH535 administrated groups showed an increase in cleaved Caspase-3 staining. Results confirmed that treatment with NVD encouraged apoptosis as the dead cells number amplified in a concentration-dependent manner (Fig. 10b, c). Western blot data demonstrated more cleavage in NVD treated group in contrast to control (Fig. 10a).

RETRACTED

**Fig. 10:** NVD and FH535 administration induces apoptosis in HCT116 xenograft tumors in athymic nude mice. **a** Effect of NVD and FH535 treatment (15 and 25 mg/kg) on protein expression of cleaved Caspase 3 of HCT116 implanted xenografts tumors in athymic nude mice. **b**, **c** Immunohistochemistry of cleaved Caspase 3 of NVD and FH535 administrated tumor xenograft vs untreated control tumor xenografts. The data are representative of three independent experiments with similar results

#### NVD and FH535 baskets propagation in xenograft tumors

Cyclins are a family of dogmatic proteins that systematize the advance of the cell cycle. Cyclins make active cyclin-dependent kinases (CDKs), which manage cell cycle processes through phosphorylation. Dysregulation of cyclin D1 gene expression or function contributes to the loss of normal cell cycle control during tumorigenesis. Immunoblot analysis illustrated downregulation of cyclin D in NVD and FH535 treated group (25 and 15 mg/kg) as compared to a control group. A marked difference was observed among NVD, FH535 treated (25 and 15 mg/kg) and control in an expression of cyclin D in immunohistochemistry analysis (Fig. 11a, b).

**Fig. 11:** NVD and FH535 hamper proliferation in xenograft tumors in athymic nude mice. **a** Effect of NVD and FH535 administration (15 and 25 mg) on protein expression of cyclin D of HCT116 implanted xenograft tumors in athymic nude mice. **b** Immunohistochemistry of cyclin D tumor xenograft vs untreated control tumor xenografts. Data are presented as the mean ± SD. **P < 0.01 (Scale bar, 100 µm). The data are representative of three independent experiments with similar results

#### NVD and FH535 administration diminish β-catenin and survivin expression in xenograft tumors

Effect of NVD and FH535 (15 and 25 mg/kg) on β-catenin and survivin expression in HCT116 xenograft tumors was corroborated by immunoblotting, immunohistochemical staining, and RT-PCR. An outstanding sink in expression was seen. The xenograft tumors (HCT116) revealed inclined levels of β-catenin protein. The dose-dependent effect of NVD and FH535 on HCT116 xenograft tumors confirmed an outstanding sink in β-catenin and survivin protein intensity at 2.5 and 1.25 mg doses (Fig. 12a). A prominent decrease in β-catenin expression in NVD and FH535 treated group in contrast to control group was seen by immunohistochemical staining of HCT116 xenograft tumors in athymic nude mice (Fig. 12b). To explore, either the experimental decrease in β-catenin protein was owing to decreased transcription of *β*-*catenin* gene, alteration of β-catenin expression by NVD induction in HCT116 xenograft, a marked decrease in mRNA expression by employing RT-PCR, was observed to be in dose dependent manner. At 15 and 25 mg/kg of NVD, a significant decline in β-catenin expression was observed (Fig. 12c).

RETRACTED

**Fig. 12:** Effect of NVD and FH535 administrated on HCT116 xenograft tumors for protein expression. **a** Expression of Akt, β-Catenin and Survivin protein by immunobloting in NVD administrated and control group, experiment performed in triplicate. **b** Effect of NVD and FH535 administrated on protein expression of β-Catenin and control as detected by immunohistochemical staining. Data are presented as the mean ± SD. **P < 0.01. (Scale bar, 100 µm). **c** Effect of NVD on expression of mRNA of β-Catenin by RT-PCR

#### NVD and FH535 inhibits Akt phosphorylation in HCT116 xenografts in athymic nude mice

Akt and β-Catenin signaling pathways are a vital watchdog in cell proliferation, differentiation, and growth. AKT phosphorylation encourages β-Catenin transcriptional activity and hence AKT and β-Catenin association plays a vital role in tumor progression and invasion. The HCT116 xenografts administrated with NVD and FH535 in a dose-dependent approach buckets AKT phosphorylation. Immunoblotting showed down regulation of AKT protein expression by administration of NVD and FH535 (15 and 25 mg/kg), which in turn hampers proliferation. The control and treated groups illustrated prominent differences in AKT protein expression (Fig. 12a).

## Discussion

The chief herald lesions for CRC are adenomas, and a meta-analysis of the occurrence of adenomas among U.S. adults has anticipated a range from 22% to over 50%, with a pooled frequency of approximately 30% [23]. Among individuals in whom an adenoma has been spotted and detached, 10–15% per year will go on to develop another, recurrent, adenoma [24]. Consequently, probing the role of vitamin D in colorectal adenoma frequency and recurrence provides significant information concerning its prospective position for thwarting colorectal malignancies during the earlier steps in the carcinogenesis pathway.

HCT116 and HT29 cells consequent from human colorectal adenocarcinoma at the metastatic stage are a generally used cell model for advanced metastatic colorectal cancer, which presently have no efficient alleviate. A perfect therapeutic loom is to develop drugs that are confined to aim tumors while scanting normal tissues.

RETRACTED

Moreover, the studies working with breast cancer, lung cancer, prostate cancer, squamous cell carcinoma (SCC) illustrated that 1α, 25(OH)_2_D_3_ or vitamin D analogues, showed a prominent anticancer effect. This effect of 1α, 25(OH)_2_D_3_ and its derivatives, acts through the VDR to control proliferation and apoptosis. The study related to SCC cells revealed that treatment of 1α,25 (OH)_2_D_3_ induces G0/G1 cell-cycle arrest because of the transcriptional activation of CDKN1B subsequent pRb hypophosphorylation [25–29].

Reports revealed that treatment of 1α, 25(OH)_2_D_3_ downregulates BCL2 expression in MCF-7 breast tumor and HL-60 leukemia cells and increase protein expression of BAX and BAK in prostate cancer, colorectal adenoma, and carcinoma cells. Also 1α,25(OH)_2_D_3_ has exposed to standardize protein expression of BCL2 family and illustrated that 1α,25(OH)_2_D_3_, might trigger caspase effector molecules [30]. Keeping all effects of VD in view we formulated protein-vitamin D-pectin nano-emulsion (NVD) to explore its anticancer activity.

Cellular propagation consequential in tumor pattern might occur due to the alteration in cell cycle regulation [31, 32]. A vital primary origin of cancer succession is recognized to speedy and candid propagation results to series and expansion of tissue accrual. Results of MMT assay specified that NVD is definite in its activity and efficient against cell cancer cell lines from different derivation. Cell growth in both HCT116 and HT29 cells is altered by NVD. Treatment with NVD resulted in the arrest of cellular proliferation in a concentration-dependent approach; magnification in the hammering of cell viability was experiential with amplifying in the concentration of dose.

P21 and p27, as members of the Cip/Kip family, have general structures and activities. Their mechanisms for cell cycle reticence may differ. In the current study, appraisal of apoptosis encouraged in HCT116 and HT29 cells demonstrated that NVD is extremely competent inducers of apoptosis in dose-dependent manner. Also our study revealed downregulation of Cyclin B1, D1, A and E, and Cdk-2, 4 and 6 expression and accompanied upregulation of cdk inhibitors WAF1/p21 and KIP1/p27 expression in NVD treated cells. In addition, NVD administrated CRC cells demonstrated arrest in the G2 phase of the cell cycle. These results are momentous since cell cycle regulation is a fundamental target for expectancy against CRC.

PARP, a characteristic caspase substrate, is a central player of DNA repair against environmental stress and in the prolongation of cell viability. Cleavage of PARP is a feature of apoptosis [33]. PARP cleavage ensues concomitantly with cleavage of procaspase 3, 7, and 9 in a concentration-dependent manner, signifying that NVD encouraged apoptosis in HCT116 and HT29 cells is mediated in the course of an central apoptosis pathway.

RETRACTED

Frequent studies have demonstrated that PARP-1 is overexpressed in various human tumors  [34–36]. Besides, it was exhibited that PARP-1 take crucial part in colon cancer expansion [37, 38] since its expression was noticeably elevated in colon cancer and was allied with tumor size and histopathology  [38]. Above results reinforced our results revealing elevated expression of PARP in NVD administrated cells in contrast to control.

Bcl-2 family connections are the principal overseer of apoptosis. Their overexpression stalwartly hampers apoptosis owing to cytotoxic injuries by the eradication of free radicals, preclusion of mitochondrial passage pattern, and the liberation of cytochrome c [39, 40]. Bcl-2 known as an apoptosis suppressor which is upstream effector in the cell death network is extremely expressed in a most of human malignancies. A heterodimer complex is formed by bax and Bcl-2 consequently deactivate the proapoptotic effects of the bax [41]. Hence, the expression levels of these apoptotic proteins were assessed in this study. Bcl-2 and Bcl-xL, the anti-apoptotic proteins, illustrated downregulated expression in NVD treated cells as compared to control cells in dose-dependent manner. The pro-apoptotic proteins, Bax and Bak, pro-apoptotic proteins, showed upregulated expression in NVD administrated HCT116 and HT29 cells in contrast to control cells. Hence our study anticipated that NVD arbitrated incline in the expression of Bax and down regulation of Bcl2 expression possibly will be potent route through which NVD induces apoptosis in CRC. Furthermore, NVD showed potential to target Bcl-xl and Bak signifying its pleiotropic effect on the apoptotic signaling pathway.

Studies illustrated that phosphorylation of β-catenin at Ser552 by protein kinase AKT results to its amplified transcriptional activity [42] and also revealed that overexpression of both a constitutively dynamic and a dominant negative form of AKT had analogous effects to those originate with the wild-type and dominant negative types of CK2α, respectively [43]. In Present study, AKT and β-catenin illustrated downregulated expression by treatment of NVD in HCT116 and HT29 CRC cells in contrast to control cells. Immunofluorescence staining of HCT116 and HT29 cells confirmed a downregulation in p-Akt expression and β-catenin at a concentration of 60 µM of NVD administrated in contrast to control. Momentous Alexa fluor staining of p-akt (cytoplasm) of both cell lines (green fluorescence) were pragmatic in control, whereas the expression of p-Akt as specified by staining was significantly diminished in NVD treated cells. Additional current data demonstrated that NVD induction of HCT116 and HT29 cells resulted in apoptosis through reticence of β-catenin and p-Akt. While FH535 β-catenin inhibitor baskets Akt phosphorylation which in turn reduces β-catenin protein expression. NVD treatment to β-catenin inhibitor induced cells auxiliary augmented diminishes of β-catenin expression, supporting the fact that these modifications are arbitrated by protein kinase B (Akt). Our data support the involvement of AKT in encouraging the transcriptional activity of β-catenin and also proposed that CK2a may be involved in this event. Sustaining this involvement, studies have illustrated that CK2 hyper triggers AKT by phosphorylation at Ser129. Captivatingly, mutation of Ser129 to alanine results in a prominent decline in catalytic activity of AKT in vivo and also declined phosphorylation of Thr308 in vitro [44].

RETRACTED

The results obtained in our study support a mechanism of CK2α-dependent regulation of β-catenin transcriptional activity that may bypass the negative complex formed by axin/APC/GSK3b, but it still deems numerous phosphorylation steps. One occurs at residue Thr393 of β-catenin by CK2 in a region of the ARM domain where APC interrelates to encourage β-catenin deprivation [45, 46]. The phosphorylation may be carried out by CK2α subunit alone and probably in the nucleus where the CK2α have been detected and also, remarkably, where APC interrelates with β-catenin to encourage its nuclear export [47]. Our study also supports a mechanism of CK2α dependent up-regulation of β-catenin transcriptional activity and cell viability arbitrated by phosphorylation of AKT. Conversely, this is an essential event for such regulation, because further phosphorylations may be also crucial. Akt being the most decisive downstream effector of CK2 and phosphatidylinositol 3 kinase (PI3-K). Once triggered by phosphorylation, AKT encourages cell endurance through hampering pro-apoptotic proteins [48]. The initiation of PI3K/Akt can prompt the canonical Wnt signaling during the phosphorylation of GSK-3β by the phosphorylated Akt1/2, blocking the pattern of β-catenin destroying complex (28). Consequently, the upregulation of PTEN may basket the canonical Wnt signaling by activating the deficit of β-catenin. Whereas present data revealed that treatment of NVD to HCT116 and HT29 colon cells decreases the phosphorylation of PI3 k, AKT and diminished the protein expression of β-catenin. Recently it was demonstrated that the effect might not be from the decreased phosphorylation of GSK-3β by PTEN/PI3 K/Akt cascade. As it is susceptible to mutation of β-catenin in HCT116 cells, the β-catenin can’t be marked by the destruction complex in this colon cancer cells [49]. Additional we examined that treatment of NVD inhinit the mRNA expression of β-catenin. Thus our study stalwartly demonstrated that NVD has convincing anti-proliferation activity in human colon cancer cells, encouraging apoptosis and the anti-proliferation effect of NVD may be mediated by PI3 K/Akt signaling by blocking Wnt/β-catenin signaling transduction, through inhibiting the β-catenin expression respectively.

RETRACTED

Because of critical roles in crucial cellular processes, including the homeostasis, growth control, and regeneration of cells, the two signaling pathways, Wnt/β-catenin and RAS-ERK must be firmly synchronized [50–52]. Unusual activations may lead to types of cancer including CRC.

The communication between Wnt/β-catenin and RAS/ERK pathways has been confirmed. Studies illustrated that RAF-1-MEK-ERK pathway is instantaneously triggered by recombinant Wnt3a administration in NIH3T3 and L cells, specifies direct relations of the Wnt/β-catenin and RAF-1-MEK-ERK pathways [53]. The P13K and ERK are too triggered by Wnt3a, and that is allied with cellular propagation [54, 55]. Auxiliary numerous observations have been confirmed control of the RAF-1-MEK-ERK signaling cascade by the Wnt/β-catenin signaling [56–58]. Additionally, GSK3β, chief player of Wnt/β-catenin pathway, is controlled by RAS-MAPK and PI3 K-Akt signaling cascades, and the cross-talk between GSK3β and RAS-MAPK or PI3K/AKT/mTOR signaling pathways is implicated in the pathogenesis of HCC and pancreatic cancer [59, 60]. These observations support our results illustrating patent reticence of MAPK i.e. ERK ½ phosphorylation, that could be a potential mechanism for NVD mediated cell death and apoptosis in HCT116 and HT29 cells.

Earlier study has proved that overexpressed β-catenin can actually interact with NF-κB indirectly and hamper its activity, signifying a narrative mechanism for β-catenin-mediated oncogenesis; namely, β-catenin hampers NF-κB activity, which may permit cancer cells to flee immune scrutiny and also the study stalwartly proposed that β-catenin is a chief mediator for the cross regulation of NF-κB by the GSK-3β pathway [61]. The commencement of NFκB entails phosphorylation; results demonstrated that the transcription factor was not triggered due to inhibition of its phosphorylation by NVD which in turn results in hampering of cancer cell endurance. These observations recommended that inactivation of NFκB via inhibition of its phosphorylation at p65 P-Ser529 might be one of the mechanisms by which NVD induce growth arrest in HCT116 and HT29 cells.

RETRACTED

An observation illustrated that the significant interaction and proficient inhibition of NF-κB by β-catenin in colorectal cancer cells involves phosphatidylinositide 3-kinase (PI3 K) [62]. Impediment of PI3 K by chemical inhibitors overturns the pattern of β-catenin and NF-κB protein complexes. In dormant colorectal cancer cells, β-catenin and NF-κB are confined in the cytoplasm, and treatment with PI3K inhibitor results to nuclear translocation of NF-κB and membrane retention of β-catenin. On the contrary, it is veiled whether PI3K directly serves as an alliance player between β-catenin and NF-κB or alternatively plays a role in β-catenin-arbitrated suppression of NF-κB set off by diverse stimuli. Present data suggested that reticence of overexpression of β-catenin by treatment of NVD in HCT116 and HT29 results in decreased protein expression of NF-κB and PI3 K, hence this may be one of the potential mechanism cell death and apoptosis.

Genetic deviation in the JAK/STAT/SOCS-signaling pathway emerges to be allied with a colon as well as a rectal cancer risk. The JAK/STAT/SOCS-signaling pathway has a vital part in immune defense and control of inflammation specified its indispensable association with cytokine signaling. Furthermore, the machinery of the pathway, such as STAT3, is involved in promoting uninhibited cell growth and survival in the course of dysregulation of gene expression responsible for apoptosis, cell-cycle regulation, and angiogenesis [63]. JAK1, JAK2, and STAT3 have been allied with colorectal cancer development [64]. In addition of commencement of NFκB, there is an incentive of assorted other pro-survival pathways during series of cancer, including MAPK (ERK, JNK) and STAT3, usually not hampered by proteasome inhibitor therapy in tumors or cell lines. Any drug affecting numerous pathways might be used as an efficient chemotherapeutic [65]. CK2 is also compulsory for cytokine and growth hormone prompted incentive of the JAK-STAT signaling pathway so we assume that inhibition of CK2 catalytic subunit may be accountable for hampering JAK-STAT signaling pathway in colorectal cancer. Conversely, in HT29 cells, JAK2 protein expression was appreciably hampered with a prominent alteration in STAT3 phosphorylation, hence we assume that may be a potential mechanism for NVD arbitrated cell death and apoptosis in HT29 cells.

Survivin (BIRC5), an allies of the inhibitor of apoptosis (IAP) protein family, is a allot anti-apoptotic protein which enhances tumor cell growth [66]. Survivin is copiously expressed during fetal growth in humans but is infrequently there in adult tissues [67], though, most human cancer cells articulate survivin, including colorectal cancer cells and CRC cells express up to 68% as reported [68]. Studies also revealed that survivin expression allies with advanced disease, shoddier endurance, and chemotherapy and radiation confrontation [69, 70]. Hence, survivin is of emergent concern as a possible beneficial target to hinder cancer rise [71]. Survivin boosts tumor proliferation by revamping various momentous cell signaling pathways. Our results evidently revealed remarkable reticence of an anti-apoptotic protein survivin expression in both HCT116 and HT29 cells by treatment of NVD. Therefore NVD is predictable to provide more influential potential to restrain tumor incursion and metastasis, representing as a novel tool for potential future CRC treatment.

RETRACTED

We confirmed related finding in in vivo system, Athymic mice implanted with HCT116 xenografts with NVD and FH535 β-catenin inhibitor, administration induced a dose-dependent downregulation of β-catenin, surviving, and Akt phosphorylation. Akt is a crucial element of signaling cascades for cell strength and propagation throughout growth and series of malignancy. Currently, protein expression of β-catenin, Survivin, and FH535 β-catenin inhibitor p-Akt was assessed in NVD and FH535 administrated against an untreated control group.

Our results displayed, for the foremost time, the in vivo potential of NVD and FH535 in reducing the HCT116 xenograft expansion. In tissue specimens from xenografts, the decreased expression of *β*-Catenin, and down-regulation of Cyclin D1 and caspase 3 cleavage symbolize an encouraging validation of the NVD and FH535 potential in vivo in tumors inhibition and present adequate direct confirmation for the reticence of the canonical Wnt/*β*-Catenin pathway and of *β*-Catenin target genes by NVD and FH525 in human CRC. Results demonstrated stimulation of p-Akt protein and cyclin D expression in the control group as compared to both groups encouraged with NVD and FH535 administration. The decline in protein expression is in support of reticence of propagation in groups by NVD and FH525 administration. A Manifest discrepancy was present between expressions of p-Akt and cyclin D in control verses NVD and FH535 administrated group when checked by staining (Immunohistochemistry). The expression of Cyclin D and p-Akt was downregulated in NVD and FH535 administrated group as contrast to the control group. The decline in tumor growth and volume with a simultaneous decrease in β-catenin and survivin proteins expression levels were seen in the NVD and FH535 administrated groups by western blot analysis, may have various therapeutic significance. Further mRNA expression was checked by RT-PCR, revealed a decline in β-catenin gene expression in NVD and FH535 group as compared to control. The conclusion of the current observation can have a constructive suggestion and translational impact to colorectal cancer subjects as it demonstrates that NVD can affect tumor succession, which could amplify the continued existence and superiority lifespan of the subjects suffering from colorectal carcinoma.

RETRACTED

Furthermore, the conclusion of the current study is that the NVD hold ability for maturity as a possible therapeutic and chemopreventive agent against colorectal cancer. While auxiliary experiments are considered necessary to entirely scrutinize the association of NVD with Wnt/*β*-Catenin pathway, we suppose that to attain significant clinical results in the treatment of colorectal cancers harboring a stabilizing mutation of *β*-catenin, NVD could symbolize a superior prospect to amplify the efficacy of therapies.

The present study proposed that NVD act as an inhibitor of the Wnt/β-catenin pathway has the prospective to restrain tumor invasion and metastasis in both in vitro (HCT116 and HT29 cells) and in vivo (Xenograft) CRC models: NVD demonstrated evident and constant reticence of colorectal cancer cell proliferation. This prospective to restrain CRC invasion and metastasis were evident by cell cycle regulators and apoptotic proteins (Pro apoptotic and ant apoptotic proteins). The anticancer effect of NVD has been recognized to the inhibition of β-catenin and AKT protein expression. Additionally to this, we observed that NVD diminish the expression of an anti-apoptotic protein survivin. Survivin encourages tumor proliferation by way of modulating multiple critical cell signaling pathways. Consequently, NVD is predictable to offer more powerful prospective to restrain tumor invasion and metastasis, representing as a promising strategy for future CRC treatment.

Based on our finding, we recommend a mechanism by which NVD elicits its effect on CRC. We chiefly took under consideration different pathways like Wnt/β-catenin, Erk and PI3K/Akt. As reported NVD decrease protein expression of β-catenin, AKT and also reduces protein expression of survivin, the downstream target of Wnt/β-catenin signaling, consequently, we proposed that NVD may act as a β-catenin inhibitor.

## Additional file

**Additional file 1.** **Figure S1.** A) Mice weight was taken twice weekly and values represent mean±SD of six mice. **, p < 0.02 (25 mg/kg),*, p < 0.01 (15mg/kg) vs control group;**, p < 0.001. (B) H&E staining of kidney brain, heart, liver and lung of NVD treated mice vs. control for toxicity studies. **Table S1**. Slide review: preliminary observations.

RETRACTED

## Abbreviations

NVD: vitamin D-Nanoemulsion
CRC: colorectal cancer
CSCs: cancer stem cells
DMSO: dimethyl sulfoxide
DMEM: Dulbecco′s Modified Eagle′s
PI: propidium iodide
DAPI: 4′,6-diamidino-2-phenylindole, dihydrochloride
DAB: diamminnobenzidine
VDR: vitamin D receptor
µM: micro molar
EGF: epidermal growth factor
EGFR: epidermal growth factor receptor
IGFBP: IGF-binding proteins
DMEM: Dulbecco’s Modified Eagle’s Medium
FBS: fetal bovine serum
PBS: phosphate buffer saline
MTS: mano-thermo-sonication
PARP: poly (ADP-ribose) polymerase
